# A Novel Medical Image Denoising Method Based on Conditional Generative Adversarial Network

**DOI:** 10.1155/2021/9974017

**Published:** 2021-09-28

**Authors:** Yuqin Li, Ke Zhang, Weili Shi, Yu Miao, Zhengang Jiang

**Affiliations:** ^1^School of Computer Science and Technology, Changchun University of Science and Technology, Changchun 130022, China; ^2^Zhongshan Institute of Changchun University of Science and Technology, Zhongshan, China

## Abstract

Medical image quality is highly relative to clinical diagnosis and treatment, leading to a popular research topic of medical image denoising. Image denoising based on deep learning methods has attracted considerable attention owing to its excellent ability of automatic feature extraction. Most existing methods for medical image denoising adapted to certain types of noise have difficulties in handling spatially varying noise; meanwhile, image detail losses and structure changes occurred in the denoised image. Considering image context perception and structure preserving, this paper firstly introduces a medical image denoising method based on conditional generative adversarial network (CGAN) for various unknown noises. In the proposed architecture, noise image with the corresponding gradient image is merged as network conditional information, which enhances the contrast between the original signal and noise according to the structural specificity. A novel generator with residual dense blocks makes full use of the relationship among convolutional layers to explore image context. Furthermore, the reconstruction loss and WGAN loss are combined as the objective loss function to ensure the consistency of denoised image and real image. A series of experiments for medical image denoising are conducted with the denoising results of PSNR = 33.2642 and SSIM = 0.9206 on JSRT datasets and PSNR = 35.1086 and SSIM = 0.9328 on LIDC datasets. Compared with the state-of-the-art methods, the superior performance of the proposed method is outstanding.

## 1. Introduction

The appearance of noise is random and inevitable, which is closely related to image quality assessment. Since the radiation-sensitive property of medical images, various noises occur during the acquisition process, especially when radiation dose reduces. As a fundamental step of image processing, image denoising needs to remove the noise and preserve image details. In general, image denoising methods can be divided into two categories: traditional methods and deep learning methods, including local and nonlocal methods [1].

The common traditional methods deal with noise according to various filters. Discrete wavelet [2, 3] with simple structure and fast calculation is one of the popular traditional filter-based denoising algorithms. For nonlocal filter-based algorithms [4–6], Zhang et al. employed nonlocal means-based regularization to measure noise artefacts [5]; Dabov et al. proposed a strategy of block matching and 3D transform-domain collaborative filtering (BM3D) [6]. Since the mentioned methods are limited to noise diversities, a list of parameters is selected for model optimization, such as the kernel size in the median filter [7], the searching window definition and weight in the nonlocal means methods [8], the regularization parameters in the total-variation minimization [9], and the parameters in the Gaussian filters [10]. In fact, in the process of image restoration, the related prior knowledge of noise is difficult to obtain.

With the development of deep learning, some methods have outperformed traditional image analysis and computer-aided diagnosis technologies. Deep learning methods work well for uncertain noise types robustly with their outstanding ability of high-level feature representation. Deep convolutional neural networks have made great achievements in the field of image denoising such as deep convolutional neural network (DCNN) [11]. The network of DnCNN [12] is an extension of DCNN with residual learning strategy for removing Gaussian noise. Deep learning methods have already applied to medical imaging denoising, such as convolutional neural network denoising autoencoder (CNN DAE) [13]. At present, generative adversarial network (GAN) achieves great progress for image denoising with a min-max two-player game between the generative network and the discriminator network [14, 15]. Nevertheless, as an unconditional generative model, the samples generated by GAN in the training process cannot be controlled and lack diversity [16]. To meet this challenge, the conditional generative adversarial network (CGAN) is proposed by Mirza et al. [17], which can be regarded as an extension of basic GAN. Specifically, CGAN feeds additional information to a generator and discriminator with different modalities and controls the generative model with conditional variable. The advanced research methods based on conditional generative adversarial networks (CGAN) [18] are employed for image denoising, owing to its advantage of conversion of image characteristics. Kim and Lee [1] used CGAN for low-dose chest image denoising. Zhang et al. [19] proposed an image denoising model based on deep convolution neural network and combined the batch normalization and residual learning for noised X-ray images. Chen et al. [20] presented a two-step framework of GAN-CNN to remove unknown noise. Compared with lossless images, the restored images have a certain degree of loss in details and structural changes.

In this paper, a novel medical image denoising method based on CGAN is proposed. Different from traditional CGAN, the proposed method contributes to preserving image context relationship and structural information. It is well known that super-resolution reconstruction can improve the quality of images and recover the details. To make full use of the information and relationship of each layer in CGAN, some residual dense blocks (RDBs) are embedded in the generator, which are used for superresolution reconstruction. The noise image and its corresponding gradient image are merged as conditional information to input into the proposed model, which enhanced the noise information in noise image. In addition, the reconstruction loss and WGAN loss are combined as the objective loss function.

Here are main contributions of this paper:

1. This work introduces a novel medical image denoising method based on CGAN, which contributes to preserving image context relationship and structural information
2. We construct a super-resolution generator by embedding some residual dense blocks (RDBs), which makes full use of the information and relationship of each layer in CGAN
3. In this paper, the noise image and its corresponding gradient image are integrated as conditional information to input into the network. By this way, the noise information is enhanced. Besides, this paper employed a structural hybrid loss comprising reconstruction and WGAN losses to train the model efficiently
4. In order to verify the performance of the proposed method, ablation experiments and comparison experiments are conducted on JSRT and LIDC datasets. Besides, the residual images and two indicators are employed to evaluate the denoised images. Simulation results demonstrate that the proposed model achieves higher performance while preserving more structural and contrast information

To clearly describe and demonstrate the proposed method, this paper is organized as follows: Section 2 provides the architecture of our model. In Section 3, some related experiments are conducted to verify the performance of the proposed model. Finally, Section 4 shows the conclusion of this paper.

## 2. Methods

### 2.1. Modelling for Image Denoising

Noise reduction for medical images in this paper can be modelled as follows. Let *x* ∈ ℝ^*N*×*N*^ represent a noise image, and *y* ∈ ℝ^*N*×*N*^ is the corresponding normal image. Usually, the relationship between *x* and *y* can be formulated as

(1) $$\begin{array}{c} x=\sigma \left(y\right). \end{array}$$

The task of noise image denoising is to find a function *f* to satisfy

(2) $$\begin{array}{c} \arg\underset{f}{\min}{\left\|y-f\left(x\right)\right\|}_{2}^{2}. \end{array}$$

The purpose of the denoising process is to find an adaptive function *f* and map the noise image to a normal image. This optimization problem can be solved by different objective functions with different models.

### 2.2. Foundation and Overview

Generative adversarial network (GAN) [21] as a powerful tool of generative model has been introduced to image denoising. As shown in Figure 1(a), basic GAN is divided into two parts, the generator network *G* and the discriminator network *D*. The generator *G* tries to produce a synthetic sample according to the real data distributions, which usually come from low-dimensional random noise. The discriminator *D* with the output of a score plays a role of classification between a synthetic sample and real sample. The generator tries to deceive the discriminator with an optimization method, while the discriminator is trained to distinguish synthetic samples from the real samples. Therefore, a GAN is such a game process: if *G* generates a sample and gets a high score in *D*, which proves that *G* is trained well, and if *D* can distinguish easily between the synthetic and real samples, the effect of *G* is insufficient. This pair of networks trained alternately until the samples generated by *G* is almost indistinguishable from the real samples. Mathematically, the process of the game between *G* and *D* can be formulated as a two-player minimax game as

(3) $$\begin{array}{c} \underset{G}{\min}\underset{D}{\max}E_{x∼P_{\text{data}}}\left[\log\left(D\left(x\right)\right)\right]+E_{z∼P_{\left(z\right)}}\left[\log\left(1-D\left(G\left(z\right)\right)\right)\right], \end{array}$$

where *P*_data_ and *P*_(*z*)_ are the distributions of real sample and synthetic sample, respectively. *D*(*x*) denotes the probability which *x* subjects to the real data, and *z* is the random noise which is used as the input of *G*.

In order to guide the generation of GAN, the conditional GAN (CGAN) is introduced [17]. As shown in Figure 1(b), CGAN is an extension of GAN with conditional information integrated in both the generator and discriminator. By this way, CGAN can generate the desired samples. The process of the game can be formulated as

(4) $$\begin{array}{c} \underset{G}{\min}\underset{D}{\max}E_{x∼P_{\text{data}}}\left[\log\left(D\left(x\left|y\right.\right)\right)\right]+E_{z∼P_{\left(z\right)}}\left[\log\left(1-D\left(G\left(\left.z\right|y\right)\right)\right)\right], \end{array}$$

where *y* is condition information.

Both the basic GAN and the CGAN methods can recover noise image and improve the quality in vision, while they ignore the image structure preserving. Medical images illustrate the location, appearance, and relationship of tissues and lesions, which are obliged to accurate diagnosis and treatment. In general, the type of noise is always unknown for image denoising. Especially, a lot of quantum noise and some other kinds of noise are commonly generated in medical image acquisition. Therefore, medical image denoising is required to maintain the consistency of both vision and content between the recovered image and the real image. Inspired by this, we proposed a novel medical image denoising method based on CGAN.

The overall architecture of the proposed network is designed as in Figure 2. In the overall architecture, *G* has 4 convolution layers and 6 residual dense blocks (RDBs) which extract abundant context features to generate a synthetic (denoised) image close to the real image. Each convolution layer has a Leakey ReLU after instance normalization. Then, *D* with the fully connected layer maps the feature vector to a confidence value to distinguish synthetic image and real image in terms of structure consistency. Some modules in the proposed framework will be introduced in the following subsections.

### 2.3. Gradient Enhancement for Noise Image

Different from traditional algorithms, the proposed method employs a mechanism that incorporates gradient information. In this work, the noise image and its corresponding gradient image are merged as conditional information to input into the proposed model. In the noise images, one noise point is always different from the surrounding pixels. Hence, the gradient information will be larger than normal pixels.

To calculate the image gradient, we need to compute the gradient for each pixel in an image. The image can be regarded as a two-dimensional discrete function. The image gradient is actually the derivation of this two-dimensional discrete function as

(5) $$\begin{array}{c} M\left(x,y\right)=\sqrt{{\left(gx\right)}^{2}+{\left(gy\right)}^{2}}, \end{array}$$

where *gx* and *gy* are the horizontal gradient and vertical gradient, respectively. *gx* and *gy* can be formulated as Equations (6) and (7), respectively.

(6) $$\begin{array}{c} gx=\frac{\partial f\left(x,y\right)}{\partial x}=f\left(x+1,y\right)-f\left(x,y\right), \end{array}$$

(7) $$\begin{array}{c} gy=\frac{\partial f\left(x,y\right)}{\partial y}=f\left(x,y+1\right)-f\left(x,y\right). \end{array}$$

By calculating the gradient on each pixel, the gradient map is obtained as in Figure 3.  Figure 4 illustrates the process of gradient enhancement for noise image. The green boxes denote different operations in the previous image. Firstly, the corresponding gradient map is acquired by calculating the gradient for each pixel in an image. Meanwhile, the texture and edge information in an image is obtained. Secondly, taking information such as edges and textures into account, thresholding approach is used in gradient maps. That is to say, the points lower than the threshold in the gradient image are considered as edges and texture structures. In this research, the median of the gradient image is set as the threshold. Then, we will obtain a new gradient image. Intuitively, these two gradient maps are represented by histograms as shown in Figure 4. Finally, the noise image is enhanced by adding up the noise image and the corresponding new gradient image.

### 2.4. Residual Dense Block

Developing efficient and adaptive denoising models with prominent structure preserving plays an important role in medical imaging, which helps clinicians accurately interpret medical images. In addition, it facilitates improving the ability of feature recognition in medical images. Some studies have shown that the application of image restoration methods based on ResNet is helpful to the preservation of organs and fine structural details [22].

The residual dense network (RDN) was firstly proposed by Zhang et al. for image superresolution [23]. More previously, Lim et al. employed residual blocks to build a wider network which was called EDSR [24]. Ma et al. used 5 residual blocks in the generator of GAN for low-dose CT image denoising [25]. Tai et al. used memory block to construct MemNet [26]. With the depth of network increasing, the features in each convolutional layer would be hierarchical with different receptive fields [23]. Nevertheless, these methods stack building blocks in a chain way, which ignores the information from each Conv layer. In view of this, Zhang et al. proposed residual dense block (RDB) to make full use of the information and relationship of each layer [23].

In this research, the superresolution reconstruction that can improve the quality of images and recover the detail is considered. To make full use of information in each convolutional layer, a super-resolution method is employed to the generator network. In this paper, the generator with 6 residual dense blocks (RDBs) is utilized to extract the context information among layers. The structure of RDB is designed as in Figure 5; the contiguous mechanism is implemented by connecting the state of preceding RDB to each layer of current RDB directly. In this way, not only the feed-forward nature is preserved, but also the rich local features are extracted efficiently. Therefore, the output of *n*th Conv layer of *d*th RDB is formulated as

(8) $$\begin{array}{c} F_{d,n}=\text{ReLU}\left(W_{d,n}\left[F_{d-1},F_{d,1},\cdots ,F_{d,c-1}\right]\right), \end{array}$$

where *F*_*d*−1_ and *F*_*d*_ are the input and the output of the *d*th RDB, respectively. *W*_*d*,*n*_ is the weight of the *n*th convolution layer.

### 2.5. Loss Function

The definition of loss function is critical for the performance of GAN-based image denoising method. To a great extent, the loss function of deep learning influences the noise image restoration process [25]. Many researchers studied different image denoising models by employing various loss functions. The mean squared error (MSE) or L2 loss function is the most widely used for many GAN-based models [14, 15, 24]. However, it includes the regression-to-mean problem, which causes oversmoothing and texture information loss. Furthermore, with the introduction of the networks of VGG-16 and VGG-19 pretrained on ImageNet, the perceptual loss was proposed to cope with the problems caused by MSE [27–29]. In this paper, we conduct some experiments with perceptual loss, and the performance of the results is poor. To effectively deal with various noises and preserve image structure, a structural loss integrates reconstruction loss and WGAN loss and is defined as the final objective loss function.

#### 2.5.1. Reconstruction Loss

Some previous studies have found that it is beneficial to introduce a more traditional loss to the GAN objective [18, 29]. As we all know, L1 and L2 distances are the most commonly used loss functions in regression tasks. Furthermore, it is reported that the L2 loss function may result in blurring [18]. Therefore, this research employs the L1 distance as the reconstruction loss rather than L2, which is constructed with *ℒ*1-norm and formulated as

(9) $$\begin{array}{c} L_{\text{Recon}}={\left\|I_{\text{raw}}-G\left(I_{\text{noise}}\right)\right\|}_{1}, \end{array}$$

where *I*_raw_ is the original raw image and *I*_noise_ is the image with artificial noise.

#### 2.5.2. WGAN Loss

The above reconstruction loss focuses on structure preservation but ignores image details. To conquer this dilemma, a WGAN loss is added to provide detailed information.

On the basis of standard GAN loss, WGAN loss [30] introduces Wasserstein distance instead of JS divergence as the additional condition to measure the difference between synthetic and real distributions. Besides, the usage of Wasserstein distance improves a better measurement between the ground-truth image and the denoised image, which can mitigate the problem of gradient vanishment and accelerate the network convergence effectively.

The process of the game between *G* and *D* also can be formulated as a two-player minimax game as

(10) $$\begin{array}{c} \underset{G}{\min}\underset{D}{\max}E_{x∼P_{\text{data}}}\left(D\left(x\;\;|\;\text{ y}\right)\right)-E_{z∼P_{\left(z\right)}}D\left(G\left(z\;|\;y\right)\right). \end{array}$$

With Wasserstein distance and conditional information, the WGAN loss can learn a generative model which can fit the distribution of the real samples and prevent overfitting effectively. In Equation (10), this paper integrates the noise image and its corresponding gradient image as conditional information as in Section 2.3. Once the augmented image is conducted as conditional information, the denoised images will be outputted. Therefore, the objective function of Equation (10) can be rewritten as

(11) $$\begin{array}{c} L_{\text{W}‐\text{GAN}}=\underset{D}{\max}E\left[D\left(x\right)-D\left(x^{\prime }\right)\right], \end{array}$$

where *x* = {*I*_grad_aug_, *I*_raw_}, *x*′ = {*I*_grad_aug_, *I*_denoised_}, *I*_grad_aug_ is the augmented image, *I*_raw_ is the original raw image, and *I*_denoised_ generated by the generator *G* denotes the denoised image.

#### 2.5.3. Final Loss Function

During the training process of the model, the total loss between the normal image and the denoised image is computed, which can be back-propagated for the proposed model to update the parameters. The final structural loss function of the proposed network consists of reconstruction loss *L*_Recon_ and WGAN loss *L*_W‐GAN_, defined as

(12) $$\begin{array}{c} \underset{G}{\min}\underset{D}{\max}L_{\text{W}‐\text{GAN}}\left(D,G\right)+\lambda_{1}L_{\text{Recon}}\left(G\right), \end{array}$$

where *λ*_1_ is a hyperparameter.

## 3. Results and Discussion

### 3.1. Dataset and Evaluation Indicators

#### 3.1.1. Dataset

In the experiments, the raw X-ray images from the public Japanese Society of Radiological Technology (JSRT) dataset [31] were adopted, consisting of 246 PA chest radiographs collected from thirteen Japanese institutions and one American institution. In addition, we added various unknown artificial noises including Gaussian noise, salt and pepper noise, and some random noise to the chest X-ray images to generate 246 pairs of images with the resolution of 256∗256. Some example images from the adopted dataset are illustrated in Figure 6.

Another dataset used in this paper was the Lung Image Database Consortium and Image Database Resource Initiative (LIDC-IDRI or LIDC) [32]. The LIDC dataset is a web-accessible international resource, which is commonly used for diagnosis, detection, and classification of lung nodules. This dataset consists of 1018 subjects of thoracic, and it is annotated by 4 radiologists. The resolution of each slice of the CT is 512∗512, and the thickness of each slice ranges from 0.6 to 5.0 mm. For the experiments, we adopted the first 2 patient ids (LIDC-IDRI-0001 and LIDC-IDRI-0002) comprising of 394 CT slices. Furthermore, we added various unknown artificial noises including Gaussian noise, salt and pepper noise, and some random noise to the chest X-ray images to generate 394 pairs of images with the resolution of 256∗256. Some example images from the adopted dataset are illustrated as Figure 7.

#### 3.1.2. Evaluation Indicators

The experimental results were evaluated in terms of peak-signal-to-noise ratio (PSNR) and structural similarity index (SSIM). These two indicators were defined as in Equations (13) and (14), respectively.

(13) $$\begin{array}{c} \text{PSNR}=10\log_{10}\left(\frac{{\left(2^{n}-1\right)}^{2}}{\text{MSE}}\right), \end{array}$$

(14) $$\begin{array}{c} \text{SSIM}\left(X_{1},X_{2}\right)=\frac{\left(2\mu_{X_{1}}\mu_{X_{2}}+C_{1}\right)\left(2\sigma_{X_{1}X_{2}}+C_{2}\right)}{\left(\mu_{X_{1}}^{2}+\mu_{X_{2}}^{2}+C_{1}\right)\left(\sigma_{X_{1}}^{2}+\sigma_{X_{2}}^{2}+C_{2}\right)}, \end{array}$$

where MSE was the mean square error between two image patches. *μ*_*X*_1__ and *μ*_*X*_2__ were the sample means of patch *X*_1_ and patch *X*_2_, respectively. *σ*_*X*_1__^2^ and *σ*_*X*_2__^2^ denoted the sample variances of patch *X*_1_ and patch *X*_2_, respectively. *σ*_*X*_1_*X*_2__ was the crosscovariance between the two image patches; *C*_1_, *C*_2_ were the stable constants. When *X*_1_ and *X*_2_ were more similar, the value of SSIM was closer to 1.

### 3.2. Parameter Settings

As the foundation of the proposed method, the images with random artificial noise were used as the condition of the CGAN to input into the network. For the super-resolution generator, 6 residual dense blocks (RDBs) were embedded in, to make full use of the information in each convolutional layer and extract the context information among the convolutional layers. Different from the traditional conditional GAN, image patches were extracted. The proposed method cut the input into the image patch with the size of 70∗70 at random. In addition, the integration of Wasserstein distance and *ℒ*1-norm was employed as the objective loss function. The hyperparameters were set as follows: *λ*_1_ was 0.5, batch size was 1, learning rate was 2*e*-3, and epoch was 1500.

In the training stage, a pair of images from the training set were inputted to both the generator and discriminator, where the generator would produce a denoised image and the discriminator would map the image into a confidence value. With the method of Adam, the generator would be optimized to produce a better result of denoised image which should be close to the ground truth to earn the confidence of the discriminator. Finally, the trained network tested the test noise images and output the denoised results. The overall process of the proposed algorithm is described in Algorithm 1.

### 3.3. Ablation Analysis

#### 3.3.1. Residual Dense Blocks

Generally speaking, the methods based on super-resolution reconstruction can improve the quality of images and recover the details. The 6 residual dense blocks (RDBs) were used for superresolution reconstruction in the generator in this paper. To prove its superiority, an ablation experiment without residual dense block (RDB) was implemented on the JSRT dataset. By adding some unknown noise to the dataset, the SSIM of each result is shown in Figure 8; some denoised examples are shown in Figure 9. From Figures 8–9, we can see the advantage of RDBs in image super-resolution reconstruction; the method with RDBs can keep details and remove noise to a large degree.

#### 3.3.2. Gradient Enhancement

In conditional GAN, the noise image and its corresponding gradient image were integrated as conditional information to input the network in this paper. In noise images, the isolated noise is different from the surrounding pixels; therefore, its gradient will be larger than normal pixels. Besides, the method of thresholding was adopted to ignore the edge and texture information in the gradient maps. Therefore, adding gradient information is beneficial to enhance noise in theory. To test our idea, this paper also made an ablation experiment without gradient enhancement. In this experiment, only the noise image was adopted as conditional information for comparison. The superparameter epoch was set as 500; the coefficient of reconstruction loss was 0.5. The denoised results are shown in Figure 10 in which the evaluation of PSNR and SSIM was listed. The method with gradient enhancement achieved satisfying results.

#### 3.3.3. Objective Loss Function

Previous studies have proved that reconstruction loss can focus on structure preserving, but at the same time, it also ignores the image details. Moreover, the WGAN loss attempts to learn a generative model, which is aimed at fitting the distribution of the real samples and preventing overfitting effectively. As a result, the WGAN loss is added to supplement detailed information for reconstruction loss in this paper.

From some ablation experiments with different objective loss functions, we found that perceptual loss will damage the structural information in images, which is described in Section 3.4, and the proposed method outperforms in vision and content.

### 3.4. Comparison Analysis

We compared the performance of the proposed method with several state-of-the-art methods and ablation experiments on the datasets of Section 3.1.1 for medical image denoising. As follows, Figure 11 gives the denoising results of different methods. In order to quantify the denoising results of Figure 11, this paper made residual images between the ground-truth and the denoised images. The residual image was obtained by calculating the absolute difference between the noise image and the denoised image pixel-wisely. Then, the values in residual images were normalized to interval [0-1], and the final results were visualized as shown in Figure 12. The values of pixels closer to 1 indicate that the denoising results are poor and change the structural information of image. To further verify the denoising results of different methods, PSNR and SSIM were adopted to evaluate the performance.

In Figure 11, Figure 11(a) illustrated the synthetic noise image with various unknown artificial noises. This paper implemented the method of [27], which integrated Wasserstein distance and perceptual loss as the objective loss function on the basic conditional GAN. By comparing on the same experimental dataset setting, the denoising results are shown in Figure 11(c). On this basis, we used the basic GAN loss instead of Wasserstein distance and combined it with the perceptual loss; the results are shown in Figure 11(d). The method by combining the basic GAN loss and reconstruction loss which was proposed by Zhang et al. [33] was implemented in this paper; the denoising results are shown in Figure 11(e).  Figure 11(f) shows the denoising results by the proposed method which used the sum of Wasserstein distance and reconstruction loss as the objective loss function.

From the comparative experiments of Figure 11, it is obvious that the details of (c) and (d) are visually clearer than others. Then, we quantified the denoising results of each group of experiments by making residual image between denoising result and ground truth. The residual image was obtained by calculating the absolute difference between the noise image and the denoised image. The residual images of Figures 11(c) and 11(d) are visualized in Figures 12(a) and 12(b), respectively. Both the denoised images of Figures 11(c) and 11(d) severely damaged the structure of the image.

The residual images of Figures 11(e) and 11(f) are shown in Figures 12(c) and 12(d), respectively. Figures 11(f) and 12(d) are the denoised results of the proposed method in this paper. From Figures 12(c) and 12(d), it can be seen that the effect of denoising of Figure 11(e) was lower than the proposed method. Moreover, our method worked best in terms of structure and contrast preservation.

Figure 11 shows some denoised samples by various methods, and the Figure 12 illustrates the residual images between the denoised image and the noise-free image. From Figure 11, all methods removed most of the noise. However, Figure 12 reveals that the proposed method preserved more structural details and displayed better defined contrast. Furthermore, it would be of great significance for the field of medical image analysis. Therefore, we can infer that the objective loss function with perceptual loss will affect the structural information in the process of denoising. And our method achieved a better effect than other comparative experiments.

Table 1 displayed the performance evaluation about the denoising results based on ground truth with different methods. The performance of the results was measured by PSNR and SSIM indicators. The SSIM evaluation revealed the similarity between the experimental results and the ground truth. The PSNR values illustrated the quality of the processed images compared to the ground-truth. From Table 1, it was clear that the noise images had relatively low SSIM and PSNR because they were damaged by some specific distribution of noise on the ground truth. Since the restored images removed noise effectively, SSIM and PSNR were improved slightly. Ledig et al. [28] proposed a SRGAN model based on generative adversarial network by combing adversarial loss and perceptual loss. The first three denoising methods took perceptual loss as a part of their objective loss function. We also implemented these three denoising methods on JSRT and LIDC datasets. In this research, the feature extractor was a 19-layer VGG network consisting of 16 convolutional layers and followed by 3 fully connected layers. The outputs of the 16th convolutional layer of VGG were extracted as features in the perceptual loss function. However, the first three denoising methods obtained poor performance. Therefore, combined with the results of Figures 11 and 12, we can conclude that the methods with perceptual loss destroyed the original structure in images and caused lower mean PSNR and mean SSIM about image quality. Reference [33] combined GAN loss and L1 loss to train the model. Zhong et al. [14] used DenseNet CNN as the generator network and employed WGAN loss and L2 loss as its objective loss function. From Table 1, these comparative methods cannot achieve a satisfactory performance for medical image denoising. The proposed method achieved the best performances in quantitative analysis and also reduced the noise to a large degree. Finally, we can conclude that our method removed the noise successfully while preserving structural and contrast information of the images, and our proposed method was promising for practical applications.

## 4. Conclusions

We develop a novel medical image denoising model based on conditional GAN. Instead of focusing on the complex network structure construction, this paper is dedicated to image context exploration and structure preservation. Firstly, a generator with super-resolution reconstruction is used to improve the quality of denoised image against other generators. Secondly, different from traditional denoising GAN models, this paper combines the noise image with its corresponding gradient image as conditional information of conditional GAN, which enhanced the noise information. Thirdly, the model is trained based on residual calculation by combining synergistic loss functions so that the denoised results are as close to the ground truth as possible. Finally, residual images and evaluation indicators are used to quantify the denoised results on JSRT and LIDC datasets. Compared with different denoising models, the proposed model not only improves the quality of denoised images but also maintains the detailed structure consistent with the lossless images.

## Figures and Tables

**Figure 1:** The architecture of the basic GAN and conditional GAN.

**Figure 2:** Overall framework of the proposed model (INorm indicates instance normalization; LReLU denotes Leakey ReLU).

**Figure 3:** Some examples of noise images and their corresponding gradient maps.

**Figure 4:** The process of gradient enhancement for noise image.

**Figure 5:** Architecture of the residual dense block (RDB).

**Figure 6:** Some examples selected in the JSRT dataset.

**Figure 7:** Some examples selected in the LIDC dataset.

**Figure 8:** Evaluation the quality of denoised image with SSIM. The green line represents without RDBs.

**Figure 9:** Examples of denoising results: (a) ground truth; (b) noise images with unknown noise; (c) denoised results without RDBs; (d) denoised results with the proposed method.

**Figure 10:** (a) Is ground truth; (b) is noise images; (c) is the method only with noise image as conditional information; (d) denotes the results of our proposed method.

**Figure 11:** Some generative denoised results by different methods: (a) noise image; (b) ground truth; (c) WGAN+perceptual; (d) perceptual+CGAN; (e) L1+CGAN; (f) the proposed method.

**Figure 12:** Residual images between comparative experiment and ground truth: (a) denotes Figures 8(c) and 8(b); (b) represents Figures 8(d) and 8(b); (c) indicates Figures 8(e) and 8(b); (d) shows Figures 8(f) and 8(b).

**Algorithm 1:** The training process of the proposed medical image denoising method based on conditional generative adversarial network.

**Table 1:** Average PSNR and SSIM of the denoised images by different denoising models on the JSRT dataset.

Methods	PSNR (mean)		SSIM (mean)	
	JSRT	LIDC	JSRT	LIDC
Noise	15.4436	18.3036	0.1170	0.1390
WGAN+perceptual [27]	16.3217	20.1425	0.7635	0.7930
CGAN+perceptual	12.5834	18.3698	0.4420	0.6326
SRGAN [28]	16.2250	21.4650	0.7779	0.8023
CGAN+L1 [33]	32.6180	34.1577	0.8945	0.8936
Zhong et al. [14]	32.9856	33.0452	0.8960	0.8847
The proposed method	33.2642	35.1086	0.9206	0.9328

## Data Availability

Data used in this paper's preparation was obtained from the JSRT and LIDC-IDRI datasets (http://db.jsrt.or.jp/eng.php, https://link.springer.com/article/10.1007/s00330-015-4030-7?gclid=EAIaIQobChMI3eupq97d8gIVFauWCh0vyQYAEAAYASAAEgJ01fD_BwE).

## References

[1] Kim H. J., Lee D. (2020). Image denoising with conditional generative adversarial networks (CGAN) in low dose chest images. *Nuclear Instruments and Methods in Physics Research Section A: Accelerators, Spectrometers, Detectors and Associated Equipment*.

[2] Mondal T., Maitra M. (2014). Denoising and compression of medical image in wavelet 2D. *International Journal on Recent and Innovation Trends in Computing and Communication*.

[3] Mustafa N., Khan S. A., Li J. P., Khalil M., Kumar K., Mohaned G. Medical image de-noising schemes using wavelet transform with fixed form thresholding.

[4] Buades A., Coll B., Morel J. M. A non-local algorithm for image denoising.

[5] Zhang H., Ma J., Wang J. (2015). Statistical image reconstruction for low-dose CT using nonlocal means-based regularization. Part II: an adaptive approach. *Computerized Medical Imaging and Graphics*.

[6] Dabov K., Foi A., Katkovnik V., Egiazarian K. (2007). Image denoising by sparse 3-D transform-domain collaborative filtering. *IEEE Transactions on Image Processing*.

[7] Liu H., Zhou N. An improved filtering algorithm based on median filtering algorithm and medium filtering algorithm.

[8] Salmon J. (2010). On two parameters for denoising with non-local means. *IEEE Signal Processing Letters*.

[9] Beck A., Teboulle M. (2009). Fast gradient-based algorithms for constrained total variation image denoising and deblurring problems. *IEEE Transactions on Image Processing*.

[10] Shih Y. T., Chien C. S., Chuang C. Y. (2012). An adaptive parameterized block-based singular value decomposition for image de-noising and compression. *Applied Mathematics and Computation*.

[11] Vincent P., Larochelle H., Bengio Y., Manzagol P. A. Extracting and composing robust features with denoising autoencoders.

[12] Zhang K., Zuo W., Chen Y., Meng D., Zhang L. (2017). Beyond a Gaussian denoiser: residual learning of deep CNN for image denoising. *IEEE Transactions on Image Processing*.

[13] Gondara L. Medical image denoising using convolutional denoising autoencoders.

[14] Zhong Y., Liu L., Zhao D., Li H. (2020). A generative adversarial network for image denoising. *Multimedia Tools and Applications*.

[15] Zhang X., Feng C., Wang A., Yang L., Hao Y. (2021). CT super-resolution using multiple dense residual block based GAN. *Signal, Image and Video Processing*.

[16] Ma R., Zhang B., Hu H. (2020). Gaussian pyramid of conditional generative adversarial network for real-world noisy image denoising. *Neural Processing Letters*.

[17] Mirza M., Osindero S. (2014). Conditional Generative Adversarial Nets. https://arxiv.org/abs/1411.1784.

[18] Isola P., Zhu J., Zhou T., Efros A. A. Image-to-image translation with conditional adversarial networks.

[19] Zhang F., Cai N., Wu J., Cen G., Wang H., Chen X. (2018). Image denoising method based on a deep convolution neural network. *IET Image Processing*.

[20] Chen J., Chen J., Chao H., Yang M. Image blind denoising with generative adversarial network based noise modeling.

[21] Goodfellow I., Abadie J. P., Mirza M. Generative adversarial nets.

[22] Kulathilake K. A. S. H., Abdullah N. A., Sabri A. Q. M., Lai K. W. (2021). A review on deep learning approaches for low-dose computed tomography restoration. *Complex & Intelligent Systems*.

[23] Zhang Y., Tian Y., Kong Y., Zhong B., Fu Y. Residual dense network for image super-resolution.

[24] Lim B., Son S., Kim H., Nah S., Lee K. M. Enhanced deep residual networks for single image super-resolution.

[25] Ma Y., Wei B., Feng P., He P., Guo X., Wang G. (2020). Low-dose CT image denoising using a generative adversarial network with a hybrid loss function for noise learning. *IEEE Access*.

[26] Tai Y., Yang J., Liu X., Xu C. MemNet: a persistent memory network for image restoration.

[27] Yang Q., Yan P., Zhang Y. (2018). Low-dose CT image denoising using a generative adversarial network with Wasserstein distance and perceptual loss. *IEEE Transactions on Medical Imaging*.

[28] Ledig C., Theis L., Huszár F. Photo-realistic single image super-resolution using a generative adversarial network.

[29] Chen L., Zheng L., Lian M., Luo S. (2020). A C-GAN denoising algorithm in projection domain for micro-CT. *Molecular & Cellular Biomechanics*.

[30] Gulrajani I., Ahmed F., Arjovsky M., Dumoulin V., Courville A. Improved training of Wasserstein GANs.

[31] Shiraishi J., Katsuragawa S., Ikezoe J. (2000). Development of a digital image database for chest radiographs with and without a lung nodule: receiver operating characteristic analysis of radiologists' detection of pulmonary nodules. *American Journal of Roentgenology*.

[32] Armato S. G., McLennan G., Bidaut L. (2011). The lung image database consortium (LIDC) and image database resource initiative (IDRI): a completed reference database of lung nodules on CT scans. *Medical Physics*.

[33] Zhang J., Guo M., Fan J. (2020). A novel generative adversarial net for calligraphic tablet images denoising. *Multimedia Tools and Applications*.

